The article "Application of Intravenous Anesthesia in Laparoscopic Hiatal Hernia Repair of Children" was retracted in 2023. Reasons: suspected computer-generated content; unreliable results or conclusions; lack of ethics approval or compliance; missing or withdrawn patient consent.

# Application of Intravenous Anesthesia in Laparoscopic Hiatal Hernia Repair of Children

**DOI:** 10.1155/2022/5290813

**Published:** 2022-06-29

**Authors:** Xueli Zhu, Haiyang Yang, Meimin Qu, Jianshe Wang, Jian Fei, Linyu Shi

**Affiliations:** Department of Anesthesiology, Children's Hospital of Nanjing Medical University, Nanjing, Jiangsu, 210008, China

## Abstract

In order to solve the stress problem in laparoscopic hiatal hernia repair of children, improve surgical safety, and reduce surgical risk, this study compared the perioperative changes of epinephrine, norepinephrine, IL-6, IL-10, and hemodynamics in children undergoing laparoscopic surgery under intravenous general anesthesia and general anesthesia combined with an epidural block. In this study, 40 children aged 1–3 years who planned to undergo laparoscopic ortopexy and those who planned to undergo laparoscopic high ligation of hernia sac, aged 23.84 1.6 months and weighed 14.9 1.1 kg, were randomly divided into general anesthesia combined with the epidural block group (group *A*) and a total intravenous anesthesia group (group *B*), with 20 subjects in each group. The results are as follows: There were no differences in age, gender, body weight, anesthesia time, pneumoperitoneum duration, and functional time between the two groups. Cytokines: Compared with *T*0, the levels of IL-6 in *T*2, *T*3, *T*4, and *T*5 groups were significantly increased (*P* < 0.01). IL-10 levels: *T*2, *T*3, *T*4, and *T*5 groups were further increased, and the difference was statistically significant compared with *T*0 (*P* < 0.01). There was no difference between groups (*P* > 0.05). The recovery time in group *B* was shorter than that in group *A* (*P* < 0.01), and the total amount of propofol and fentanyl in group *B* was less than that in group *A* (*P* < 0.01). Through research on intravenous anesthesia treatment, it has been proved that total intravenous anesthesia can relieve perioperative pressure, reduce intravenous injection, and reduce the recovery time of children. However, its effect on cytokines is not obvious, so intravenous anesthesia is the most appropriate anesthesia mode in laparoscopic hiatal hernia repair surgery, which has practical significance.

## 1. Introduction

As a minimally invasive technique, laparoscopic operation (LO) has been widely used in the surgical field due to its advantages such as less incision bleeding, less trauma, and quick post-operative recovery and has gradually changed some traditional treatment methods in pediatric surgery, as shown in Figure 1. Although a large number of studies have shown that the degree of stress caused by laparoscopic surgery is less than the conventional laparotomy, but that caused by co_2_ pneumoperitoneum intra-abdominal pressure, carbon dioxide-absorbed hypercapnia, and surgery at the end of the internal pressure drop similar ischemia and reperfusion injury factors can induce the body's stress response [1]. This can lead to changes in endocrine metabolism, triggering an inflammatory immune response. Moreover, the imbalance of homeostasis does not stop with the end of the operation, but excessive stress lasting for a certain period can change the homeostasis of the body, induce immune suppression, affect the safety and prognosis of the operation, and lead to the occurrence of perioperative complications and increased mortality. The most typical pathological change of hiatal hernia is gastroesophageal reflux and long-term reflux can cause complications such as pharyngitis and asthma. Therefore, anesthesia of such patients is a great challenge for anesthesiologists [2]. Anesthesiologists need careful preoperative evaluation and correct intraoperative management to ensure that the side effects of anesthesia can be reduced and patients can recover quickly. Hiatal hernia repair is usually performed under general anesthesia. General anesthesia commonly used in surgery includes total intravenous anesthesia (TIVA) and general anesthesia combined with dural block maintenance. Although these two general anesthesia methods can be used in this kind of surgery, but each has its advantages and disadvantages in clinical application [3]. In this study, children who underwent selective laparoscopic testicular descent fixation and high ligation of hernia sac were selected as the research subjects, and total intravenous anesthesia or general anesthesia combined with dural anesthesia were used to compare the dynamic changes of the children, and their change trend in the perioperative period and their relationship with the occurrence and development of stress response were analyzed. By comparing the effects of different anesthesia methods on stress response in the perioperative period, we screened out the anesthesia methods which can effectively reduce stress response and inhibit traumatic inflammatory reaction.

## 2. Literature Review

Likhvantsev et al. believes that since the first laparoscopic cholecystectomy was reported in 1987, laparoscopic surgery has been widely used in the field of surgery for its advantages of small trauma, safety, simplicity, and quick postoperative recovery [4]. Bhattarai and Kamal noted that with the widening of the scope of adaptation and the increase of the difficulty of laparoscopic surgery, the pathophysiological changes caused by CO_2_ pneumoperitoneum in the special working environment of laparoscopic surgery have been paid more and more attention by scholars. Although minimally invasive laparoscopic surgery alleviates the trauma to the body to a certain extent, the application of carbon dioxide pneumoperitoneum in laparoscopic surgery will still affect the changes of the internal environment of the body and produce stress response, thus exerting a certain influence on the neuroendocrine immune system of the body [5]. Abazid et al. concluded that children's response to stress is different from that of adults due to the imbalance of development of various body systems; especially in laparoscopic surgery, carbon dioxide pneumoperitoneum will have a special effect on the pathophysiology of children. Therefore, with the continuous understanding of perioperative stress response of laparoscopic surgery in children, how to let the children complete the operation in the possible physiological state is an important subject for anesthesiologists [6]. Maharani et al. noted that in pediatric laparoscopic surgery, the child was supine, the diaphragm function increased, the pulmonary functional residual capacity (FRC) decreased, and the abdominal compliance decreased. At the same time, IAP increased, the diaphragm was affected by gravity and intra-abdominal pressure, FRC decreased tidal volume and minute ventilation (MV) decreased, and the child's oxygen level was affected [7]. In addition, Lai et al. believed that pneumoperitoneum could cause disharmony of ventilatory blood perfusion, increase in IAP, decrease in FRC, and easily lead to atasis. The peritoneal carbon dioxide disperses into the blood, and the arterial blood partial pressure of carbon dioxide (PaCO_2_) increases, which can effectively maintain the respiratory function during hypercapnia respiratory acidosis. Most of them can return to the normal level within 24 hours after surgery, and the younger the age, the faster the elimination. Simple epidural anesthesia can only block the conduction of sympathetic nerve and somatic nerve injury stimulation, but cannot change the changes of inflammatory cytokines [8]. Reazaul Karim thought that epidural anesthesia did not alter the increase of inflammatory cytokines and CRP in patients undergoing esophagectomy, suggesting that extensive epidural anesthesia could not inhibit the inflammatory stress response caused by tissue injury [9]. Somuncu et al. noted that most studies show that when the anesthesia block level reaches *T*_4_, afferent impulse and sympathetic nerve activity of most stimuli can be blocked, stress response can be reduced, and C-reactive protein (CRP) can be reduced. General anesthesia combined with epidural block anesthesia can inhibit neuroendocrine metabolism and immunity mediated by operative stress, but it cannot be completely blocked [10]. Zhao et al. said that in a comparative study of pediatric urology, he showed that the use of hemodynamically stabilizing vasoactive drugs was reduced in the epidural anesthesia combined with intravenous anesthesia group compared with the control group, possibly due to the epidural anesthesia combined with general anesthesia. Making full use of anesthesia complementarily can not only block the sensory nerve afferent stimulation in the spinal nerve root level but also can inhibit the sympathetic vagus afferent stimulation in the center by general anesthesia. This kind of central and peripheral double inhibition causes the postoperative stress response to reduce a lot obviously. At present, general anesthesia is mostly used in laparoscopic surgery for children. The application of intravenous anesthesia under general anesthesia can meet the requirements of sedation, analgesia, and muscle relaxation. At the same time, the anesthesia machine controls breathing to ensure the airway patency during surgery, which reduces the risk of reflux and aspiration in children during laparoscopic surgery and ensures the safety of surgery [11]. Zheng et al. noted that a large number of data show that general anesthesia cannot completely effectively prevent stress reactions caused by pneumoperitoneum environment and surgical stimulation, which are often manifested as increased heart rate and blood pressure, etc. In order to suppress the adverse reactions, the usual treatment is to increase the dosage of narcotic analgesics to deepen anesthesia. The increase of anesthetics will increase the burden of liver and kidney metabolism in children, and even clinically, postoperative respiratory recovery, delayed recovery and postoperative respiratory depression, and other adverse reactions often occur [12]. For this reason, Yu et al. applied general anesthesia combined with epidural block in pediatric laparoscopic surgery, intraoperative hemodynamics, changes in stress hormones, and changes in immunity and anticytokines were all altered compared with anesthesia alone. The purpose of this study was to compare the intervention of two anesthesia methods on perioperative stress response in children undergoing laparoscopic surgery, so as to provide some theoretical basis for the selection of anesthesia methods in children undergoing laparoscopic surgery [13].

## 3. Research Method

### 3.1. Research Subject Selection

Laparoscopic orchiopexy and laparoscopic pressure ligation in 40 children aged 1–33 years were ASA (American Society of Anesthesiologists) Class I-II. All the children were from the Children's Hospital affiliated to a medical university, including 29 males and 11 females, with an average age of 23.8 ± 1.6 mm and a weight of 14.9 ± 1.1 kg [14]. Preoperative examination showed no complications of the endocrine system, circulatory system, and respiratory system. Normal liver and kidney function; no hormone drugs were taken before surgery; no contraindications for epidural anesthesia; no obesity or malnutrition (body mass index above or below 95% was the normal range for this age group).

### 3.2. Clinical Grouping

Forty children with laparoscopic hiatal hernia were divided into two groups, with 20 cases in each group: group *A* combined with generalized epidural block and group *B* was given general anesthesia [15].

### 3.3. Anesthesia Method

In groups A and B, lumina sodium 5 mg/kg and atropine 0.01 mg/kg were intramuscularly injected 30 min before surgery, and 22 g–24 g indignant needle was used to puncture the dorsal hand vein or ankle vein to maintain infusion during surgery. After entering the operating room, the anesthesia machine was used to monitor the Ohmeda S/5 heart rate continuously, respiratory rate, RR, mean arterial pressure, MAP, electrocardiogram. ECG, pulse oxygen saturation, SpO_2,_ end expiration pressure CO_2_, P_ET_CO_2._

Catheterization of right external jugular vein and radial artery under midazolam 0.1 mg/kg propofol 1.5 mg/kg basic anesthesia was used to obtain blood samples and monitor blood pressure. Group *A* used the method of general anesthesia extended with epidural anesthesia, GEA. Group *B* used the method of general intravenous anesthesia GA [16].

#### 3.3.1. Epidural Block Anesthesia

Group *B* received epidural block anesthesia after catheterization. *T*_12_–*L*_1_ was selected as the puncture point. After successful puncture, a 2-3 cm epidural catheter was placed in the epidural space and a trial amount of 1.2% lidocaine (without epinephrine) was injected with 3 ml of blood and cerebrospinal fluid after suction. Five minutes later, there was no toxic reaction and total spinal anesthesia. The follow-up dose of 3–6 ml was given and the total amount of elidocaine 8 mg/kg was calculated. The block plane *T*_6_–*L*_3_ was controlled [14].

#### 3.3.2. General Anesthesia Induction

Anesthesia induction in both *A* and *B* groups was induced by intravenous injection of propofol 1 mg/kg fentanyl 5 g/kg and vecurbromine 0.1 mg/kg. After oxygen and nitrogen removal for 2 min, the two groups were intubated through the mouth with open sight, followed by Ohmeda S/5 anesthesia machine and volume control ventilation (VCV) mode [17]. Tidal volume (VT) was l0-15 ml/kg, RRl8 times/min, suction/respiration ratio (1 : *E*) = 1 : 2, oxygen flow rate was 1.5 L/min, and respiratory rate was changed to 24–30 times/min after the establishment of carbon dioxide pneumoperitoneum, and blood gas analysis was performed. The final respiratory partial pressure of carbon dioxide (P_ET_CO_2_) and airway peak pressure (P_peak_) were adjusted appropriately.

#### 3.3.3. Maintenance of Anesthesia

In both groups, a microinjection pump was used to continuously pump propofol fentanyl and vecuronium to maintain the anesthesia depth during operation [18]. The initial dose of propofol was 10 mg/kg/h, fentanyl 5 *μ*g/kg/h, vecuronium 70 *μ*g/kg/h, which were adjusted intraoperatively according to the patient's HR MAP, keeping it within 20% of the base value; The respiratory parameters were adjusted according to the change of P_ET_CO_2_, and the P_ET_CO_2_32–42 mmHg was maintained [19]. Intraoperative pneumoperitoneum pressure was maintained at 8–12 MMHG, and lactate Ringer's solution was used for venous maintenance.

#### 3.3.4. Extubation Pointer

Intravenous anesthesia was discontinued at the end of pneumoperitoneum operation in both groups. Consciousness was recovered, spontaneous breathing was recovered, respiratory rate was more than 20 times/min, protective reflex (swallowing cough reflex) was recovered, air was inhaled for 5 min, SPO2 was 95%, P_ET_CO_2_ was <50 mmHg, and the tracheal tube was removed when HR MAP was stable.

### 3.4. General Information Record

Age, weight, sex ratio, disease composition ratio (cryptorchidism/oblique inguinal hernia), operation time (disinfection ∼ application), anesthesia time (induction of anesthesia ∼ conscious extubation), pneumoperitoneum time (inflating start ∼ ventilation), and total dosage of intravenous anesthesia propofol and fentanyl were recorded in the two groups [20].

### 3.5. Respiratory and Circulatory System Indicators Were Recorded

FIR, RR, MBP, SPO2, airway peak pressure (P_peak_), and P_ET_CO_2_ was continuously monitored. These data were also recorded: 5 min before anesthesia (*T*_0_), 5 min before pneumoperitoneum (*T*_1_), 5 min after pneumoperitoneum (*T*_2_), HR, MAP, SPO2 value at the end of pneumoperitoneum 20 min after (*T*_3_) (*T*_4_), and 30 min after (*T*_5_).

### 3.6. Blood Gas Analysis Records

Blood gas analysis was performed at *T*_0_, *T*_l_, *T*_2_, *T*_3_, *T*_4_ via radial artery, and arterial CO_2_ partial pressure (PaCO_2_) PH value bicarbonate (HCO_3_) concentration was recorded.

### 3.7. Detection of Epinephrine, Norepinephrine, and IL-6 and IL-10

At *T*_0_,*T*_l,_*T*_2_, *T*_3_, *T*_4_ and *T*_5_, 5 ml of central venous blood was extracted and stored in anticoagulant tubes, respectively. We made timely use of the normal temperature low speed centrifuge 3000 turn/min for 15 min to separate plasma. We store it in a −20°C refrigerator sealed for testing. Enzyme-linked immunosorbent assay (ELISA) was conducted to measure epinephrine, norepinephrine, IL-6, and IL-10 [21]by using human blood norepinephrine kit and human blood IL-10 kit.

### 3.8. Statistical Treatment

SPSS11.0 statistical software was used for analysis and mathematical calculation. Measurement data are reported in terms of standard deviation (*X* ± *s*). Comparisons of different observations within groups were performed by identifying differences, and pial comparisons were performed by *q*-test. Comparisons between groups were performed using independent *t*-test, with *P* < 0.05 as the mean [22].

## 4. Interpretation of Result

### 4.1. The General Condition of Patients in the Two Groups

There was no significant difference between group *A* and group *B* in age, weight, gender, and disease composition (*P* > 0.05) (see Table 1).

### 4.2. Comparison of Intraoperative Conditions between the Two Groups of Children

There was no significant difference in operation time, anesthesia time (initial withdrawal of induction drug), and pneumoperitoneum time (initial increase in deflation) between the two groups (*P* > 0.05); recovery time (end of operation to awake extubation) of group *B* was significantly shorter than that of group *A* (*P* < 0.01). Intraoperative doses of fentanyl and propofol: group *B* was less than group *A*, and the difference was statistically significant (*P* < 0.01); group A did not use lidocaine (see Table 2).

### 4.3. Changes of Hemodynamics in the Two Groups

Compared with *T*_0_: after pneumoperitoneum occurred, HR and MAP in group *A* were significantly increased between *T*_2_, *T*_3_, and *T*_4_, with significant values (*P* < 0.01). MAP in group B decreased significantly at *T*_1_, and the data difference was significant compared with *T*_0_ (*P* < 0.01). There were no significant changes in other values, and the difference was not significant (*P* > 0.05). Compared with group *A*, there was no significant difference in HR and MAP at *T*_0_ between the two groups (*P* > 0.05). *T*_1_, *T*_2_, *T*_3_, *T*_4_, *T*_5_, HR, and MAP in group B were lower than those in group A, with a significant difference (*P* < 0.01). (See Table 3, Figures 2 and 3).

### 4.4. Blood Gas Analysis Was Compared between the Two Groups

Compared with before pneumoperitoneum (*T*_1_), there was no significant difference in pH values of *T*_2_, *T*_3_, *T*_4_, and *T*_5_ between the two groups after pneumoperitoneum (*P* > 0.05). Compared with group A, there was no significant change at each time point before and after pneumoperitoneum (*P* > 0.05). Compared with pre-pneumoperitoneum (*T*_l_), PaCO_2,_ HCO concentration at *T*_3_, *T*_4_ was significantly different from *T*_l_ (*P* < 0.01). Compared with group A, there was no significant difference in HCO3 concentration in *T*_3_ (*P* < 0.01), and there was no significant difference in other time content (*P* > 0.05) [23]. PaCO_2_ and HCO_3_ concentrations before and after pneumoperitoneum in both groups were within the normal range (see Table 4).

## 5. Conclusion

Stress response exists and runs throughout the perioperative period of laparoscopic surgery in children. Appropriate anesthesia can intervene and regulate the stress response. The results of this study showed that compared with general anesthesia combined with dural block anesthesia, patients in the general anesthesia group had significantly stable symptoms, no postoperative recurrence, and a lower incidence of nausea and vomiting. Postoperative recovery is faster, so all-intravenous anesthesia maintenance method is more suitable for hiatal hernia repair patients. In this study, it was found that total intravenous anesthesia could accelerate postoperative exhaustion. In a study of the effects of propofol and sevoflurane on intestinal motility, it was also found that the duration of defecation and fatigue was shorter in the propofol group than in the sevoflurane group. In contrast, when studying the effects of inhalation anesthesia and anesthesia on the arteries of the gastrointestinal tract, it was found that the different anesthetics did not affect the recovery of the gastrointestinal tract, and it was not the anesthesia but other factors that affected the time, defecation, and exhalation in the perioperative period. In conclusion, all-intravenous anesthesia in laparoscopic hiatal hernia repair of neonates is a better anesthesia solution, which can be popularized in clinical practice.

## Figures and Tables

**Figure 1:** Laparoscopic surgery.

**Figure 2:** Comparison of intraoperative HR between two groups.

**Figure 3:** Comparison of intraoperative MAP between two groups of children.

**Table 1:** Comparison of general situation between two groups of children.

Group	Case load (n)	Age (month)	Weight (kg)	Sex ratio (MF)	Proportion of incidence (cryptorchid/hernia)
*A*	20	24.5±1.2	14.6±1.0	14/6	8/12
*B*	20	23.6±1.1^*∗*^	15.3±0.9^*∗*^	15/5^*∗*^	7/13^*∗*^

Compared with group *A*, *P* > 0.05.

**Table 2:** Comparison of general conditions between two groups of children during operation.

Group	Operation time (min)	Anesthesia time (min)	Pneumoperitoneum time (min)	Awakening time (min)	Fentanyl (*µ*g)	Propofol (mg)
*A*	39.4±2.5	45.3±3.2	35.7±3.3	10.7±3.3	79.2±5.3	98.6±9.6
*B*	40.2±2.6	47.2±2.9	34.2±3.7	6.9±1.1^*∗*^	54.0±4.1^*∗*^	77.1±5.6^*∗*^

Compared with group *A*, ^*∗*^*P* < 0.01.

**Table 3:** Comparison of intraoperative HR and MAP between the two groups.

Index	Group	*T*_0_	*T*_1_	*T*_2_	*T*_3_	*T*_4_	*T*_5_
HR (Time/min)	*A*	105.32±10.30	110.43±9.82^*∗*^	131.12±11.20^*∗*^	135.72±11.21^*∗*^	127.55±10.62^*∗*^	116.2±11.32
	*B*	104.41±9.21	106.32±10.41^△^	105.20±10.45^△^	106.14±9.13^△^	106.53±11.92^△^	102.30±9.46^△^

MBP (mmHg)	*A*	61.40±4.11	63.14±4.87	78.36±5.21^*∗*^	77.64±4.93^*∗*^	76.36±3.85^*∗*^	77.40±5.20^*∗*^
	*B*	62.10±4.30	56.12±3.21^*∗*^^△^	63.48±4.60^△^	63.72±4.61^△^	65.11±3.16^△^	64.10±5.32^△^

Compared with *T*_0_^*∗*^*P* < 0.01, compared with group ^△^*P* < 0.01与T_0_此较.

**Table 4:** Comparison of arterial blood gas analysis between two groups of children before and after pneumoperitoneum.

Index	Group	*T*_1_	*T*_2_	*T*_3_	*T*_4_	*T*_5_
PH	*A*	7.40 ± 0.04	7.38 ± 0.03	7.39 ± 0.06	7.42 ± 0.05	7.35 ± 0.08
	*B*	7.41 ± 0.05	7.40 ± 0.04	7.36 ± 0.07	7.42 ± 0.03	7.35 ± 0.06

PaCO_2_ (mmHg)	*A*	36.20 ± 3.72	36.81 ± 2.48	40.10 ± 3.11^*∗*^	39.65 ± 4.12^*∗*^	41.9 ± 3.20^*∗*^
	*B*	35.60 ± 2.94	36.30 ± 2.56	39.82 ± 4.15^*∗*^	40.30 ± 4.03	40.33 ± 4.01^*∗*^

HCO_3_^−^(mmol/L)	*A*	22.84 ± 2.60	22.23 ± 3.02	24.03 ± 1.61^*∗*^	23.01 ± 1.47	23.01 ± 1.60
	*B*	22.71 ± 2.21	23.20±2.73	22.70 ± 2.24△	23.00 ± 2.38	23.12 ± 2.24

^*∗*^ *P* < 0.01 compared with *T*_1_ and ^△^*P* < 0.01 compared with group *A*.

## Data Availability

The data used to support the findings of this study are available from the corresponding author upon request.
